The article "Effectiveness, safety, and patient satisfaction of carboxytherapy as an adjunctive treatment for periorbital hyperpigmentation" was published in 2024. Journal: Skin Res Technol.

# Effectiveness, safety, and patient satisfaction of carboxytherapy as an adjunctive treatment for periorbital hyperpigmentation

**DOI:** 10.1111/srt.13651

**Published:** 2024-03-14

**Authors:** Farnoosh Seirafianpour, Najmolsadat Atefi, Nazila Ghoreishi Amin, Mohammad Reza Namazi, Elham Behrangi, Aboozar Shafiei, Mohammadreza Ghassemi, Samaneh Mozafarpoor, Azadeh Goodarzi

**Affiliations:** ^1^ Razi Drug Research Center Iran University of Medical Sciences Tehran Iran; ^2^ Department of Dermatology Rasool Akram Medical Complex Clinical Research Development Center (RCRDC) School of Medicine, Iran University of Medical Sciences (IUMS) Tehran Iran; ^3^ Department of Radiology University of Southern California (USC) Los Angeles California USA; ^4^ Department of Dermatology School of Medicine Shiraz University of Medical Sciences (SUMS) Shahid Faghihi Hospital Shiraz Iran; ^5^ Skin Diseases and Leishmaniasis Research Center Department of Dermatology Isfahan University of medical Sciences Isfahan Iran

**Keywords:** carboxytherapy, CO2 therapy, dark eye circles, DECs, eye dark circles, infraorbital darkening, periorbital darkening, periorbital hyperpigmentation, trail

## Abstract

**Introduction:**

Dark under‐eye circles or periorbital hyperpigmentation constitute a prevalent and challenging cosmetic problem with diverse etiologies and types. While modifying exacerbating habits can provide partial relief for the pigmentary and vascular factors associated with this condition, and despite the abundance of available treatment options, there is currently a lack of gold‐standard evidence‐based treatments proposed for curing this disorder.

**Objectives:**

This study aimed to assess the safety and effectiveness of carboxytherapy in treating periorbital hyperpigmentation.

**Material and Methods:**

In this 4‐week single‐arm clinical trial, 20 eligible Iranian patients with symmetric periorbital hyperpigmentation received weekly intradermal carboxytherapy. The treatment involved administering 10–20 mL of CO2 at a rate of 20 mL/min and a temperature of 15°C for a duration ranging from a few seconds to 1 min. Follow‐up assessments were conducted 1 month after the final session. The primary outcome was defined as the changes in ΔE or the variations in pigmentation observed between the orbital and extra‐orbital skin before and after the trial.

**Results:**

The patients reported satisfaction with the statistically significant reduction in hyperpigmentation achieved through carboxytherapy in the lateral (*p* = 0.002), middle (*p* = 0.001), and medial (*p* = 0.001) regions of the periorbital area. The total response rate of the patients was estimated at 20%. Patient satisfaction exceeded ΔE changes, with no significant linear relationship (*p* = 0.084).

**Conclusion:**

Carboxytherapy can be proposed as an effective and safe treatment for periorbital hyperpigmentation.

**Abbreviation**
DUC: dark under‐eye circles
POH: Periorbital hyperpigmentation

## 1 INTRODUCTION

### 1.1 Background

Dark under‐eye circles (DUC) or Periorbital hyperpigmentation (POH) pose a prevalent and challenging cosmetic concern, significantly impacting the quality of life for individuals of all ages, genders, and races.^1^ Periorbital hyperpigmentation manifests with one or more of the following features: widespread and concentrated melanin deposits (hyperpigmentation), excessive or superficial subcutaneous vasculature, and shadows resulting from pseudoherniated orbital fat.^2^ Additional risk factors include racial, familial, and genetic predispositions to hyperpigmentation, allergic shiners in atopic patients, thin and semi‐transparent skin on the lower eyelids that accentuates the vascular plexus, post‐inflammatory hyperpigmentation following contact dermatitis, sleep disorders, excessive sun exposure, weight loss, addiction, smoking, and certain medications or disorders that mimic the presentations of oculodermal melanocyte or ashy dermatosis.^3^, ^4^ Idiopathic periorbital hyperpigmentation has been documented in numerous cases involving diverse skin issues.^5^ The differentiation between pigmentary causes and those associated with vasculature can be achieved through a Wood's lamp examination, utilizing polarized light in patients presenting with periorbital hyperpigmentation.^5^

The management of periorbital hyperpigmentation varies depending on its underlying cause. Treatment modalities for periorbital hyperpigmentation encompass various approaches targeting different aspects of the condition.^6^ These include:

#### 1.1.1 Topical agents

The use of phenolic or nonphenolic bleaching agents, such as hydroquinone, tretinoin, vitamin C, arbutin, and azelaic acid, is recognized for its efficacy in reducing melanin pigmentation.^7^, ^8^ These agents act by inhibiting the tyrosinase enzyme, thereby reducing the melanin content in the epidermis.^7^, ^9^, ^10^

#### 1.1.2 Chemical peels

Chemical peels, either standalone or combined with topical bleaching agents, are employed.^11^ Glycolic acid, particularly at 20%, and a combination of lactic acid (15%) with trichloroacetic acid (TCA) 3.75%, have demonstrated significant esthetic improvement in periorbital hyperpigmentation.^11^ Pre‐treatment with tretinoin and hydroquinone for 2–4 weeks is recommended for optimal results, with post‐peel demarcation minimized through priming agents.^11^

#### 1.1.3 Lasers

Noninvasive lasers targeting pigment and vascularity have gained popularity.^12^, ^13^ Laser therapies, utilizing both long‐pulsed and picosecond laser types, have been employed to address pigmentations and vascular lesions.^14^, ^15^ Q‐switched ruby laser (694 nm), Q‐switched alexandrite laser, and Nd:Yag laser (1064 nm) are utilized to treat dark circles.^12^ Studies have shown positive responses, especially with the Q‐switched ruby laser, either alone or in combination with bleaching agents.^16^ Combining topical treatments with laser therapy is often utilized to enhance overall results.^16^, ^17^

#### 1.1.4 Autologous fat transplantation

For cases related to thin and translucent lower eyelid skin, autologous fat transplantation is employed to address periorbital hyperpigmentation over the orbicularis oculi muscle.^18^

#### 1.1.5 Fillers

Hyaluronic acid gel is used for three‐dimensional reshaping of the periorbital complex.^19^ dermal fillers are effective in correcting tear trough‐associated periorbital hyperpigmentation.^20^ While patient satisfaction is high, some individuals noted darker pigmentation post‐treatment.

#### 1.1.6 Platelet‐rich plasma (PRP)

PRP has emerged as a treatment option for dark circles, demonstrating statistically significant improvement in infraorbital color homogeneity when injected intradermally.^21^

#### 1.1.7 Surgery—blepharoplasty

Blepharoplasty, particularly transconjunctival blepharoplasty, proves beneficial in eliminating dark circles caused by shadows cast by fat deposits or excess skin.^22^ Combining this with deep‐depth phenol peel simultaneously addresses hyperpigmentation and pseudoherniation of orbital fat.^22^

#### 1.1.8 Carboxytherapy

Subcutaneous injections of CO2, administered weekly over 7 weeks in the periorbital area, have shown significant improvement in fine lines and periorbital hyperpigmentation.^23^

Carboxytherapy is an innovative and noninvasive procedure involving the transcutaneous injection of CO2.^23^ Originating in 1932 at the Royal spas in France, it was initially employed to treat obliterating arteriopathies.^24^, ^25^ Hartmann et al. conducted a study demonstrating the effectiveness of serial CO2 injections in patients with intermittent claudication (Fontaine stage II).^24^ Through Doppler and Laser Doppler examinations, they substantiated the vasomotor effect of this therapy.^24^

The subcutaneous injection of CO2 induces an oxygen deficit, triggering an increase in blood flow and the release of growth factors such as vascular endothelial growth factor (VEGF).^26^ This stimulation, in turn, promotes the generation of new blood vessels.^26^ Consequently, CO2 injection exerts a positive influence on cutaneous circulation, vasomotion, and the augmentation of capillary blood flow.^27^

### 1.2 Objectives

Given the absence of gold standards for treating periorbital hyperpigmentation, this before/after clinical trial was conducted to evaluate the safety, efficacy, and tolerability of carboxytherapy in treating this condition, as well as patient satisfaction.

## 2 MATERIAL AND METHODS

### 2.1 Trial design

This single‐arm clinical trial recruited 20 patients with symmetric dark under‐eye circles (DUC), aged 20–50 years, from the laser clinic of the Rasool Akram hospital in Tehran, Iran. After providing all patients with a comprehensive briefing on the study objectives and design, they signed informed consent forms. None of the participants had a history of receiving treatments for DUC in the previous 6 months.

### 2.2 Participants

Exclusion criteria included pregnancy, lactation, intention to conceive, unilateral presentation of DUC, bleeding diathesis, active skin infections, a history of carotid artery bypass graft or heart, kidney, liver, and lung failures, systemic disorders affecting wound healing, a history of keloid formation, and Botox injections or any other procedures at the treatment site in the past 6 months. Participants were assured of their right to withdraw from the study at their own discretion or in the case of long‐lasting complications caused by carboxytherapy.

### 2.3 Intervention

Twenty eligible patients with dark under‐eye circles (DUC) participating in this 4‐week clinical trial underwent intradermal carboxytherapy once a week. A total of 10–20 mL of CO2 was injected into the orbital skin at a rate of 20 mL/min and 15° for a few seconds up to 1 min, before the emergence of skin swelling, pain, and erythema. The patients were followed up 1 month after the final session. Photographs were taken using VisioFace® 1000D (Courage‐Khazaka Electronic, Köln) before, and 1 and 5 weeks after the final session.

### 2.4 Outcomes

VisioFace was utilized to collect quantitative data on ΔE, representing the difference in pigmentation between the lateral, middle, and medial parts of the pigmented orbital skin with adjacent normal skin in the extra‐orbital area. Photographs were taken by a blinded assessor at specific time points during the study.

In colorimetry, ΔE (Delta E) serves as a measure to quantitatively express the perceptual difference in color between two samples, essentially gauging the contrast or alteration in color that contributes to an overall change in appearance. In this study, VisioFace played a crucial role in gathering quantitative data on ΔE, specifically measuring variations in pigmentation across different skin regions. This measurement is denoted by a numerical value, where a higher ΔE signifies a more noticeable shift in color. For example, if a patient exhibited dark under‐eye circles (DUC) before treatment and experienced a change in pigmentation afterward, ΔE would precisely capture the magnitude of this change. This methodology enables researchers to impartially evaluate and measure the effectiveness of treatments in terms of pigmentation reduction or color modification in the treated skin area. In essence, ΔE acts as a color difference metric employed in this study to objectively assess and analyze the efficacy of carboxytherapy in addressing dark under‐eye circles.

### 2.5 Statistical methods

Responses were scored as follows: mild (below 25%), moderate (26%–50%), good (51%–75%), and very good (over 75%). Patient satisfaction was subjectively recorded as little, moderate, good, and excellent.

Recorded side effects of carboxytherapy included burns, prolonged swelling, pruritus, erythema, pain, and eyelid blinking.

The data, expressed as descriptive statistics (mean ± standard deviation and frequency), were analyzed in SPSS 21 using the paired t‐test and one‐way ANOVA. Due to our sample size and the distribution characteristics of the data, we employed the Pearson Correlation Coefficient to assess the relationship between the recovery percentage (quantified by changes in ΔE) and patient satisfaction. The level of statistical significance was set at *p* < 0.05.

## 3 RESULTS

The present study enrolled twenty patients with dark under‐eye circles (DUC), comprising 12 females and 8 males. Participants, with a mean age of 36.5 ± 9.5 years, were categorized into age groups: below 20 years (10%), 20–30 (15%), 30–40 (50%), and over 40 (25%). The majority of patients (65%) belonged to Fitzpatrick skin type 3. Underlying disorders were not observed in 18% of the patients, while 82% of the overall patients reported some form of underlying disorder, such as a history of minor thalassemia, allergies, or thyroid disorders. As the primary outcome measure, effectiveness was assessed using ΔE to quantify changes in pigmentation at the treated site after compared to before the treatment (Figure 1).

**FIGURE 1:** Mean ΔE values for the lateral, middle, and medial parts of the eye before and after the intervention.

The ΔE diagrams demonstrated a notable decrease in pigmentation across all areas of the treated site post‐intervention (*p* < 0.05) (Table 1). As depicted in Figure 2, the treatment response, assessed through one‐way ANOVA concerning ΔE changes, revealed no significant differences among the lateral, middle, and medial parts of the eye (*p* = 0.97).

**TABLE 1:** Mean ± SD for ΔE before and after trial in lateral, middle, and medial.

Part	Mean ± SD for ΔE		95%Confidence interval for change	*T*‐value	*p*‐value
	Before	After			
Lateral	7.9 ± 3.36	6.31 ± 2.74	(−2.5, −0.67)	−3.64	0.002
Middle	6.63 ± 2.42	5.08 ± 2.24	(−2.18, −0.92)	−5.17	<0.001
Medial	6.54 ± 2.28	4.89 ± 2.22	(−2.27, −1.03)	−5.58	<0.001

**FIGURE 2:** One‐way ANOVA of ΔE before and after the trial in different parts of the eye.

Based on the ΔE, the response rate was estimated at 20% (categorized as mild). In terms of patient satisfaction with the treatment, 60% and 40% of the patients reported responses ranging from little‐to‐moderate to good‐to‐excellent.

The correlation coefficient, calculated as 0.005 between the recovery percentage based on ΔE and patient satisfaction, suggested statistically insignificant linear relationships (*p* = 0.084).

All complications, including erythema, long‐lasting swelling, and eyelid blinking (two cases each), spontaneously resolved within about a week or with the use of warm compress and massage. Given the study center's status as a tertiary general hospital, ophthalmologic consultation was initiated within a few hours of eyelid blinking onset, and patients were advised to undergo conservative care. No sustained side effects were observed during the follow‐up. Figures 3, 4, 5, 6 display the treatment results;

**FIGURE 3:** Before and after carboxytherapy in pigmented DUC (patient 1).

**FIGURE 4:** Before and after carboxytherapy in pigmented DUC (patient 2).

**FIGURE 5:** Before and after carboxytherapy in pigmented/structural DUC (patient 3), suggesting correction of puffiness.

**FIGURE 6:** Before and after carboxytherapy in pigmented DUC (patient 4).

## 4 DISCUSSION

Periorbital hyperpigmentation (POH), also known as periocular hyperpigmentation, dark circles, or idiopathic cutaneous hyperchromia of the orbital region, is a prevalent dermatological condition with a significant impact on emotional well‐being and overall quality of life.^28^, ^29^ It manifests as bilateral, homogenous brown or dark brown pigmented macules in the periocular region, influenced by factors such as pigmentation, skin thickness, and shadows due to skin laxity.^30^, ^31^ Various treatment options, including topical agents, chemical peeling, and lasers, are available for addressing excessive pigmentation causing infraorbital dark circles.^22^

Carbon dioxide injection has emerged as an effective technique for rejuvenating facial skin affected by aging and photoaging, attributed to its ability to stimulate collagen turnover and improve microcirculation, enhancing skin blood flow.^32^, ^33^, ^34^

In a split‐side clinical trial by Nofal et al., the efficacy and safety of platelet‐rich plasma (PRP) and carboxytherapy were investigated for POH treatment in 30 patients.^35^ Carboxytherapy demonstrated significant improvement in POH, outperforming PRP in terms of simplicity, effectiveness, and patient tolerance.^35^

Ahmed et al. conducted a study comparing carboxytherapy, chemical peel, and vitamin C mesotherapy for POH treatment in 45 patients, revealing no statistically significant differences in improvements among the groups.^36^ However, the mesotherapy group reported a higher frequency of burning sensations, yet exhibited significant improvement in pigmentation and satisfaction compared to carboxytherapy.^36^

In a split‐face pilot clinical trial by Assaf.H.A et al., carboxytherapy demonstrated superior efficacy compared to microneedling with topical glutathione in treating POH in 31 female patients.^37^ The results indicated greater improvement in visual analogue scale evaluations, dermoscopic assessments, patient satisfaction, and Dermatology Life Quality Index questionnaire scores with carboxytherapy.^37^

Asilian et al. compared carboxytherapy and PRP in treating POH in a clinical trial involving 21 patients, observing significant improvement postoperatively in both groups.^38^ However, insignificant differences between the two treatments were noted, possibly influenced by various factors such as technique and skin characteristics.^38^

Throughout the study duration, a gradual reduction in skin dyschromia was observed, with patients reporting diminished periorbital wrinkles and improved skin texture. Carboxytherapy, a well‐tolerated and time‐efficient procedure, exhibited promising results, warranting further validation over an extended timeframe. The minimal and temporary adverse effects underscore the potential of this approach as a valuable option for POH management.

### 4.1 Study limitations

Considering the limited number of studies conducted on carboxytherapy for DUC, the present single‐arm clinical trial employed the minimum statistically acceptable sample size to assess the efficacy and safety of this method. We recommend the use of a more robust study design in future investigations. Due to the relatively short follow‐up in the present research, we suggest the implementation of comparative randomized clinical trials with larger samples and 3−6‐month follow‐ups to thoroughly document the response rate, durability, and safety. Additionally, in this study, adverse effects or complications were determined based on patient or physician reports rather than the more comprehensive Common Toxicity Criteria for Adverse Events (CTCAE) standard method.

## 5 CONCLUSION

Carboxytherapy proved to be a compelling solution for diminishing periorbital darkness with high patient satisfaction. Significant reductions in ΔE were observed in the lateral (*p* = 0.002), middle (*p* = 0.001), and medial (*p* = 0.001) regions of the orbit. A 20% response rate was achieved across all three sites, underscoring the effectiveness of carboxytherapy. While patient satisfaction surpassed changes in ΔE, indicating insignificant linear relationships (*p* = 0.084), the procedure exhibited a commendable safety profile.

Carboxytherapy, when used alone or in combination with other therapeutic methods, emerges as an effective treatment for dark under‐eye circles (DUC). Its safety and satisfactory outcomes suggest its potential application in aesthetic medicine. Nevertheless, further research is imperative to assess the durability of treatment responses and identify potential long‐term complications.

Despite the somewhat unpredictable outcomes of carboxytherapy, influenced by factors such as settings and application methods, this promising treatment demonstrates rapid healing and improved response rates. Its versatility makes it a valuable option in various medical, cosmetic, and dermatologic conditions, especially when compared to previously unsuccessful therapies.

## CONFLICT OF INTEREST STATEMENT

The authors declared no conflicts of interest regarding the publication of the present article.

## ETHICAL APPROVAL

The present study was approved by the Ethics Committee of Iran University of Medical Sciences, Tehran, Iran (IR.SUMS.MED.REC.1397.342) in 13 November, 2018. The employed carboxytherapy device manufactured by Ronak Tajhiz Ara Company (Carbocure) was also approved by the Ministry of Health and Medical Education of Iran. The patients were assured of their right to withdraw from the study and signed informed consent forms before participation.

## CONSENT FOR PUBLICATION

Written informed consent was obtained from the patients for publishing this article with their photos. A copy of the written consent is available for review by the Editor‐in‐Chief of the journal.

## Data Availability

NA.
